The article "Empirical analysis of the impact of China–Japan–South Korea transportation infrastructure investment on environmental degradation and the validity of the environmental Kuznets curve hypothesis" was retracted in 2023. Reason: a breach of policy by an author.

# Empirical analysis of the impact of China–Japan–South Korea transportation infrastructure investment on environmental degradation and the validity of the environmental Kuznets curve hypothesis

**DOI:** 10.3389/fpsyg.2022.977466

**Published:** 2022-10-18

**Authors:** Hongbo Lu, Yuanhao Liu, Arshad Ali, Rongzhi Tian, Yuanchun Chen, Yuanwei Luo

**Affiliations:** ^1^School of Economics, Jilin University, Changchun, China; ^2^Faculty of Management and Economics, Kunming University of Science and Technology, Kunming, China; ^3^Department of Economics and Finance, Greenwich University, Karachi, Pakistan; ^4^Institute for International Strategic Studies, CCPS Central Party School, Beijing, China; ^5^Business School, Zhengzhou University of Industrial Technology, Zhengzhou, China; ^6^Guangxi University of Finance and Economics, Nanning, China

**Keywords:** road infrastructure investment, rail infrastructure investment, air infrastructure investment, environmental degradation, EKC hypothesis

## Abstract

Building sustainable and affordable transport systems is a key issue for social development and sustainable urban expansion. The study used dynamic ordinary least squares (DOLS) and fully modified ordinary least squares (FMOLS) to examine the impact of transport infrastructure investment on environmental degradation in China, Japan, and South Korea over the period 1995–2020 and the validity of the EKC hypothesis. The results show that GDP has a significant positive effect, and GDP^2^ and GDP^3^ have significant adverse effects on environmental degradation, respectively. These results confirm the validity of the inverted U shaped EKC hypothesis in selected Asian countries. Road infrastructure investment has a significant positive effect, while railway infrastructure investment has a significant adverse effect on environmental degradation. Air infrastructure investment and trade opening have a progressive and statistically significant impact on environmental pollution. Modern rail systems that run on electricity are considered less polluting, so the share of rail infrastructure investment in the transport mix can help build sustainable and safe transport systems at the city Centre and intercity levels and reduce emissions in Asian countries. Moreover, strict enforcement of the prevailing environmental conditions of trade agreements should be encouraged to reduce the increasing impact of free trade on environmental pollution.

## Introduction

The Sustainable Development Goals, which took effect in 2015, ensure environmental and economic sustainability and are a pioneering commitment to developing and advanced economies. They have an overarching strategy to narrow the conflict between environmental sustainability and economic development and improve human wellbeing. The ultimate goal of the SDGs is to build affordable, accessible, safe and sustainable transport systems for all segments of society, and to build sustainable, inclusive, resilient and safe cities and human settlements. In this regard, a key issue in the transition of cities and societies to sustainable development is the improvement of transport infrastructure (Abubakar and Aina, 2019; Moschen et al., 2019; Vaidya and Chatterji, 2020; Otamendi-Irizar et al., 2022; Ozaki et al., 2022). Not only sustainable urbanization, but sustainable economic activity is entirely dependent on improved transport infrastructure (Lafortezza and Sanesi, 2019; Ragheb et al., 2022). Modern transportation systems facilitate the flow of goods, labor, services and technology and connect the hinterland with industrial or commercial cities and ports (Rodrigue, 2020). In addition, extensive transportation facilities can reduce traffic congestion, provide individuals with medical and educational services, save time and resources, reduce distribution costs, limit monopoly power, improve market efficiency, create new jobs, and facilitate business development. Undoubtedly, strengthening transportation infrastructure is essential to achieve harmless and rapid emptying in the event of natural disasters such as forest fires, earthquakes and floods (Guth et al., 2019; Guo and Qin, 2022; Jung and Thill, 2022).

The article "Empirical analysis of the impact of China–Japan–South Korea transportation infrastructure investment on environmental degradation and the validity of the environmental Kuznets curve hypothesis" was retracted in 2023. Reason: a breach of policy by an author.

However, as with most other economic activities, nurturing transportation infrastructure creates serious environmental problems. Among other industries, transport greenhouse gas emissions (GHG) have grown significantly, with transport activities accounting for 16% of total greenhouse gas emissions in 2014. Historically, the share of transport activities in GHG emissions has been on an upward trend, and globally, the transport sector’s share of GHG emissions reached 24% (see Figure 1). Global transport emissions have increased by 2.5% annually over the past decade (Jonson et al., 2020). More likely, greenhouse gas emissions from transport activities will continue to rise due to population growth, e-commerce-related freight and private car ownership (Amatuni et al., 2020). Furthermore, energy diversification related to the transport sector remains ineffective. According to the report from Global Energy Review (2020), 92% of the final energy demand of the transportation industry is for petroleum products, while 65% of the global oil demand is for the transportation industry. Undoubtedly, the 1997 Kyoto Protocol identified transport as one of the most important sources of pollution. The goal was to reduce global greenhouse gas emissions by 5.2% by 2012 (Rayegani, 2021).

The article "Empirical analysis of the impact of China–Japan–South Korea transportation infrastructure investment on environmental degradation and the validity of the environmental Kuznets curve hypothesis" was retracted in 2023. Reason: a breach of policy by an author.

**FIGURE 1:** Global sources of greenhouse gases by 2022. The Intergovernmental Panel on Climate Change 2022.

Figure 2 shows the components of global transport GHGs, for example road transport generates nearly 74% of total transport emissions and 20% of total GHG emissions. Additionally, road construction can threaten wildlife by stimulating deforestation, erosion and animal mortality, destroying farmland and depleting water resources (Bashir et al., 2020). Thus, some researchers considered road transport among transport systems is a “draconian polluter.” In contrast, few researchers have emphasized strengthening the externalities of road transport. Investment in road infrastructure reduces environmental pollution, travel times and congestion, making freight faster and cheaper. Road investments can also limit route costs, thereby reducing traffic accidents, fatalities and injuries, and increasing the number of travel options (Anas and Lindsey, 2020; Proost and Van Dender, 2020). Native grassland plants and nesting sites next to roads are easier to maintain, another ecological benefit of road investments.

**FIGURE 2:** Global transport sector greenhouse gas emissions by 2020. International Energy Association. IEA and IPCC (2014) Summary for Policymakers.

Second, the aviation industry accounts for 13 and 2% of total transport emissions and total greenhouse gas emissions, respectively (United States Environmental protection Agency, 2022). This is quite low compared to the percentage of road transport, but arguably the threat to environmental sustainability is much higher for air transport than for road transport. Robichaud (2020) stressed that air transport threatens the atmosphere and air composition of landing sites because at high altitudes it emits half of all greenhouse gases. For example, even a short round-trip flight from London to Rome produces 234 kg of carbon dioxide per passenger, more than the annual average for 17 countries (Del Rio et al., 2022). Conversely, others see the benefits of air transport, such as the International Civil Aviation Organization (2020) arguing that humanitarian and emergency aid and relief can be delivered to impoverished or disaster-stricken areas by providing transport openings in remote areas and enabling rapid transport of important things like medical supplies and transplanted organs. Hence, the externality of the aviation industry is stronger than its contrast. The aviation industry directly or indirectly facilitates international tourism and trade, improves people’s quality of life, and generates millions of jobs around the Globe (Jones and Comfort, 2020; Alamineh, 2022). Additionally, replacing commercial aircraft with the best available technology could reduce total aviation GHG emissions by 9%. This environmentally friendly solution can be more integrated into the aviation industry than in other transport sectors. Gössling and Humpe (2020) believes that the aviation industry should not be blamed for climate change, but it contributes to greenhouse gas emissions. Furthermore, the short-term harmful effects of aviation on the environment can be reversed over time.

The article "Empirical analysis of the impact of China–Japan–South Korea transportation infrastructure investment on environmental degradation and the validity of the environmental Kuznets curve hypothesis" was retracted in 2023. Reason: a breach of policy by an author.

Compared to the value of air or road transport, rail transport is relatively low at 1.6% of total GHGs. Thus, considering rail infrastructure investment would be a greener investment in transport technology. In addition, investing in rail infrastructure to expand rail transport facilities could be a viable alternative to reducing greenhouse gas emissions and working toward meeting the requirements of the Kyoto Protocol (Hong et al., 2016). Safe transportation of more passengers and cargo through the rail system enables economies of scale. A more cost-effective solution for the entire transportation industry is to increase investment in the rail industry (Lehtveer et al., 2019; Becattini et al., 2022; Ovaere and Proost, 2022). However, ranging rail systems have some unfavorable externalities. In general, distorting the price mechanism and hindering competition in the transportation industry is the result of the monopoly created by the development of the railway system. Furthermore, the construction of a rail system may not be environmentally sustainable because it requires too many inputs, such as wood, energy, steel, and cement (Chang et al., 2019). Finally, higher noise and light pollution, forest and natural habitat destruction are the main reasons for the expansion of the railway system (Ciach and Fröhlich, 2019).

Due to rapid global urbanization, there has traditionally been an increased need for infrastructure investment to facilitate inter-city and inter-city mobility. Klohe et al. (2021) argued that by 1950, 2017, and 2050, the proportion of the world’s population living in cities will reach 33, 55, and 68% respectively. On the other hand, the realization of sustainable transport systems and SDG 11 can be achieved by nurturing transport systems, and while achieving SDG-13, 14, and 15, ecological sustainability is crucial.

In cities of East Asian countries (China, Japan, and South Korea), car ownership doubles every 5–7 years with urbanization and rising incomes. With the uncontrolled growth of motorized transport, carbon dioxide (CO_2_) emissions are increasing rapidly. Recently, transportation accounted for a quarter of global energy-related CO_2_ emissions, and this proportion is continuing to grow as expected (Asian Development Bank, 2022). The recent 2021 UN Climate Change Conference in Glasgow aims to achieve rapid, deep and sustained reductions in global carbon dioxide, and more specifically, emissions reductions necessary for the Asian transport sector to limit global warming to 1.5°C. The largest proportion of greenhouse gas emissions is carbon dioxide (CO_2_), and greenhouse gas (GHG) emissions from transportation are a key factor in global climate change. Over the past 30 years, CO_2_ emissions from the transport sector in Asian countries have risen sharply, outpacing all other sectors, and at a faster rate. At present the industrialized countries (China, Japan, and South Korea) are the main sources of transport emissions, and this proportion continuous to rise sharply. Road transport accounts for 76% of fuel emissions, mainly including four-wheelers and personal pickups, while air transport accounts for only 12% of carbon emissions (Energypedia, 2021). Sodiq et al. (2019) claim that it is difficult to create sustainable cities due to underdeveloped transport infrastructure, increased traffic congestion and fossil fuel consumption, reduced mobility and urban productivity. Thus, there is a need to improve transport infrastructure, however, these expansions are accompanied by augmented costs, such as increased mortality and environmental burden (heart disease and lung cancer mortality) and the incidence of PM 2.5 emissions from transport activities (Donaldson, 2018). Therefore, in the context of the EKC hypothesis, it is difficult to establish appropriate synergies between important parts of the SDGs due to lack of knowledge.

The article "Empirical analysis of the impact of China–Japan–South Korea transportation infrastructure investment on environmental degradation and the validity of the environmental Kuznets curve hypothesis" was retracted in 2023. Reason: a breach of policy by an author.

The main purpose of this study is to reveal the environmental impact of infrastructure investment on the transportation systems of selected East Asian countries (China, South Korea, and Japan) that have undergone rapid urbanization due to industrialization and economic growth in the context of the EKC assumption. Also determine which transport investments are environmentally friendly to achieve low pollution goals and ensure the sustainability of urban transport facilities by developing greener transport investment policies and building environmentally friendly transport technologies. These in turn will support Asian countries in achieving the Sustainable Development Goals. Second, to establish policy discussions on the integration of different SDG sub-goals, there is limited evidence in the previous literature. A key policy design to achieve these sub-goals will be to explore the impact of disaggregated transport infrastructure investments. Third, the number of studies investigating the link between transport infrastructure investment and the SDGs is limited. Investigating possible links between transport investment, and environmental degradation may help develop existing research body and inform future research directions.

The article "Empirical analysis of the impact of China–Japan–South Korea transportation infrastructure investment on environmental degradation and the validity of the environmental Kuznets curve hypothesis" was retracted in 2023. Reason: a breach of policy by an author.

## Literature review

Since the publication of the seminal work of Grossman and Krueger (1991), the economic growth–environment relationship in the context of the EKC hypothesis has gained popularity among environmentalists. Grossman and Krueger (1991) revealed the dynamic relationship between economic growth and the environment using a cubic model of 42 countries, and the results showed that there is an N-type relationship between economic growth and the environment. Since then, many studies using different econometric techniques and samples have confirmed the validity of the EKC. Studies with EKC validity include (Gokmenoglu and Taspinar, 2018; Sirag et al., 2018; Ganda, 2019; Mikayilov et al., 2019; Tzeremes, 2019; Adebayo, 2020; Alola and Ozturk, 2021; Awan and Azam, 2021; Minlah and Zhang, 2021; Murshed et al., 2021). Conversely, studies that invalidate the EKC hypothesis include (Hasanov et al., 2019; Isik et al., 2019; Dogan and Inglesi-Lotz, 2020; Koc and Bulus, 2020; Pata and Aydin, 2020; Yilanci and Pata, 2020; Alola and Ozturk, 2021; Onifade, 2022). In addition, there are several other studies showing mixed results based on different types of control variables, methods or samples used in the analysis (Atasoy, 2017; Isik et al., 2019, 2021; Gormus and Aydin, 2020; Mehmood and Tariq, 2020; Gao et al., 2021). This confirms that there is no consensus among researchers on the effectiveness of EKC.

In addition, the researchers tested the EKC hypothesis using various indicators, as well as economic growth. Linking environmental degradation with source of energy is the first part of the studies. It is agreed that increasing land use and greenhouse gas concentrations due to the depletion of non-renewable energy sources will exacerbate environmental degradation, leading to biodiversity loss and global warming (Alola et al., 2019; Belaïd and Zrelli, 2019; Abbas et al., 2020; Adedoyin et al., 2020; Anwar et al., 2021; Navare et al., 2021; Pata, 2021; Amin et al., 2022; Rahman and Alam, 2022). The environmental burden of economic activity can be mitigated through the use of renewable energy sources that reduce emission levels, increase nature’s regenerative capacity, and increase the production and consumption of eco-friendly technologies (Erdogan, 2020; Saud et al., 2020; Destek et al., 2021; Usman and Hammar, 2021; Cui et al., 2022; Dagar et al., 2022). Other indicators, such as population density, that have economic as well as political or sociological implications for environmental management processes were also used in the study (Thomson et al., 2020; Vinichenko, 2021; Styhre et al., 2022). Likewise, institutions and urbanization are other indicators that have economic and social implications for environmental management (Charfeddine and Mrabet, 2017; He et al., 2018; Azam et al., 2021; Yasin et al., 2021). The debate on these topics continues among researchers, and no consensus has yet been reached.

The article "Empirical analysis of the impact of China–Japan–South Korea transportation infrastructure investment on environmental degradation and the validity of the environmental Kuznets curve hypothesis" was retracted in 2023. Reason: a breach of policy by an author.

Studies have used sources of economic activity such as agriculture, industrialization, foreign direct investment, and human capital accumulation to investigate environmental degradation. Human capital accumulation can reduce environmental pollution by raising environmental awareness (Çakar et al., 2021; Du et al., 2022). Although at each income level, the impact of human capital may vary and does not reduce environmental degradation (Tiwari et al., 2022). Free trade regimes may trigger consumption and production activities that promote environmental degradation (Nathaniel et al., 2020; Isik et al., 2021). Whereas, the increase in trade volume helps boost economic growth to cross the EKC turning point. Therefore, environmental degradation can be reduced through the contribution of the free trade regime (Sirag et al., 2018). In the early stages of foreign direct investment (FDI) inflows, the transfer of polluting industries leads to environmental deterioration, but in the long run, the transfer of environmentally friendly technologies can offset the exacerbating effect of foreign direct investment (Marques and Caetano, 2020; Christoforidis and Katrakilidis, 2021). Arguably, FDI has no statistically significant effect on environmental quality, as highlighted by Shobande and Ogbeifun (2022). Moreover, environmental pollution can be increased with industrialization as consensus by many researchers (Li et al., 2020; Singh et al., 2020; Wang Z. et al., 2020). In addition, many studies have shown that agriculture has a promoting effect on environmental pollution (Feng et al., 2018; Su et al., 2020; Ghimire et al., 2021; Miceikiene et al., 2021), whereas, limited research suggests that the role of agriculture in environmental pollution is on a downward trend (Giller et al., 2021).

Currently, discussions on the relationship between infrastructure investment and the environment continue, focusing on the relationship between transport infrastructure and environmental degradation. Erdogan (2020) published the impact of transport system infrastructure investment on environmental degradation in 21 OECD countries. Empirical results show that railway infrastructure has a significant negative impact, while road and aviation infrastructure has a significant positive impact on environmental degradation. Sun et al. (2019) empirically explore the impact of roads on air pollutant emission intensity using a city-level dataset for the period 2003–2015. The results show that road infrastructure reduces China’s pollution emission intensity and promotes green growth. Similarly, Xie et al. (2016) estimated the environmental impact of transportation infrastructure in 281 cities in China from 2003 to 2013 using a spatial Durbin model. The results show that transportation infrastructure has an adverse direct impact on the urban environment. Another study by Sun et al. (2019) selected 28 cities with subways in China and used quarterly data from 2013 to 2016 to compare the improvement effect of road renovation and the substitution effect of rail transit construction on air quality. The empirical findings demonstrate that urban rail construction has a better marginal effect on air quality cultivation. Georgatzi et al. (2020) employed dynamic ordinary least squares (DOLS) and fully modified ordinary least squares (FMOLS) techniques to explore the relationship between road and rail infrastructure investment and the environment in 12 European countries. The resulting report showed that road and rail infrastructure investments had no impact on environmental degradation.

The article "Empirical analysis of the impact of China–Japan–South Korea transportation infrastructure investment on environmental degradation and the validity of the environmental Kuznets curve hypothesis" was retracted in 2023. Reason: a breach of policy by an author.

Wang C. et al. (2020) examines the impact of transport infrastructure (rail and road) on economic growth in countries along the Belt and Road using cross-country panel data from 2007 to 2016. The results of the analysis show that the transportation infrastructure (rail and road) of countries along the “Belt and Road” plays an important role in promoting economic growth. Another study by Muvawala et al. (2021) used autoregressive distributed lag (ARDL) techniques to examine the impact of road transport infrastructure investment on economic growth in Uganda. ARDL’s empirical findings show that road transport infrastructure investment has had a significant positive impact on Uganda’s short- and long-term economic growth. Likewise, Vlahinić Lenz et al. (2018) empirically estimated the impact of transport infrastructure on economic growth in Central and Eastern European Member States (C.E.M.S.) over the period 1995–2016. Results displayed a positive impact on investment in aviation infrastructure and road infrastructure, but rail infrastructure appeared to have a negative impact on economic growth.

The literature on the relationship between transport infrastructure investment and the environment is immature, and few researchers are involved. An integral part of SDG-11 is the initiation of sustainable transport systems, and at the heart of the SDGs themselves is ensuring ecological sustainability. However, the existing literature does not show any consensus among researchers on the impact of investment in transport infrastructure on environmental degradation. Thus, the immunity of policymakers to formulate policies for harmonizing the SDGs is not satisfactory. The main purpose of this study is to fill the above literature gap by investigating the impact of disaggregated transport infrastructure investment on environmental degradation in East Asian economies (China, Japan, and South Korea) using the FMOLS and DOLS strategies for the period 1980–2020. Designing transport investment policies through empirical findings may be critical to building modern transport systems and is an important component of sustainable cities.

The article "Empirical analysis of the impact of China–Japan–South Korea transportation infrastructure investment on environmental degradation and the validity of the environmental Kuznets curve hypothesis" was retracted in 2023. Reason: a breach of policy by an author.

## Theoretical framework, development of model, and data

Ecological modernization theory (EMT) and compact city theory (CCT) are the two main theories that can be used to explain the relationship between transport infrastructure investment and the environment. Ecological modernization theory (EMT) pays particular attention to the process of social transformation through industrialization and urbanization (Saidi and Hammami, 2017; Erdogan, 2020; Nyumba et al., 2021). Accelerating the process of industrialization is also accompanied by an acceleration of social transformation. The growth of urban populations inevitably requires investment in infrastructure, including transportation. This practice may create ecological problems, such as using more resources and destroying ecological parts of urban facilities. At the same time, CCT pointed out that the demand for highly developed urban facilities, such as housing, developed and efficient transportation systems, production and consumption facilities, can be initiated by compact urbanization with high population density. Improving infrastructure by pioneering technologically efficient and advanced transportation systems can reduce energy consumption in transportation and resource use, thereby reducing environmental pollution (De Souza et al., 2018; Koh et al., 2020). Building on these theoretical backgrounds, this study uses disaggregated transport infrastructure investment and customary economic variables to explore the environmental impact of transport investment. Furthermore, after establishing the seminal work of Grossman and Krueger (1991), trade openness became an integral part of the EKC estimate (Erdogan et al., 2020; Ahmad et al., 2021). Therefore, to avoid misspecification bias, this study uses trade openness as a control factor.

The article "Empirical analysis of the impact of China–Japan–South Korea transportation infrastructure investment on environmental degradation and the validity of the environmental Kuznets curve hypothesis" was retracted in 2023. Reason: a breach of policy by an author.

Based on the above discussion, the following logarithmic model is developed to explore the impact of transport infrastructure investment on environmental degradation in East Asian countries (China, Japan, and South Korea) during the period 1995–2020.


$${\text{lnCO}}_{2\,i\,t}=\alpha_{0}+\alpha_{1}\,{\text{lnRA}}_{\text{it}}+\alpha_{2}\,\text{lnROit}+\alpha_{3}\,{\text{lnAI}}_{\text{it}}+$$

$$\alpha_{4}\,{\text{lnGDP}}_{\text{it}}+\alpha_{5}\,{\text{lnGDP}}_{\text{it}}^{2}+\alpha_{6}\,{\text{lnGDP}}_{\text{it}}^{3}+$$

(1) $$\alpha_{7}\,\text{TOPit}+\varepsilon_{\text{it}}$$

Where CO_2_ means carbon dioxide is a comprehensive indicator of environmental degradation. RA, RO, and AI denote railway infrastructure investment, road infrastructure investment, and air infrastructure investment, respectively. GDP stands for gross domestic product and TOP indicates trade openness. Furthermore, GDP^2^ is GDP squared, GDP^3^ is GDP raised to the third power. α_0_ is the intercepts, α_*i*_, indicate the factor coefficients, and i, t and ε_*it*_ represent the country, time period, and error term, respectively. GDP^3^ is included in the model to test the N-shaped EKC hypothesis for selected countries. Following the N-type EKC theory, GDP has a progressive effect on CO_2_ emissions, reflecting the increase in emissions during the initial period of growth. GDP^2^ should show adverse effects, indicating a reduction in emissions after the first turning point, GDP^3^ should show positive signs as emissions spur growth again.

The validity of the EKC hypothesis in the selected East Asian countries, whether it is U-shaped or N-shaped, can be tested considering the parameters to be estimated below.

κ_3_ > 0, κ_4_ < 0, EKC validity has an inverted U shape

κ_3_ < 0, κ_4_ > 0, EKC effectiveness is U-shaped

κ_3_ > 0, κ4 < 0 and κ5 > 0, EKC validity is N-shaped

This study mainly focuses on empirically examining the links between transport infrastructure investment and carbon emissions in selected East Asian countries (China, Japan and, South Korea) from 1995 to 2020. The measurements and descriptions of all variables are clearly highlighted in Table 1. Carbon dioxide (CO_2_) emissions are reported in millions of tones (Mmt), gross domestic product (GDP) in constant 2015 US dollars, and trade openness (TOP) in percent of GDP. The data on these variables were being obtained from the World Development Indicators (WDI), publicly available on the World Bank website. Data for air, road and rail come from the OECD database (OECD, 2020). The OECD website publishes data on infrastructure investment in the transport sector in current euro values, so we converted the euro values to current dollars using the annual average EUR/USD exchange rate published by the European Central Bank (2020). Next, using the deflator published by the World Bank (2020), we convert the current dollar value to a constant 2015 price. However, keep in mind that the World Bank’s published deflator base year varies by country, so to avoid biased estimates, we converted the deflator base year for selected countries to 2015.

The article "Empirical analysis of the impact of China–Japan–South Korea transportation infrastructure investment on environmental degradation and the validity of the environmental Kuznets curve hypothesis" was retracted in 2023. Reason: a breach of policy by an author.

**TABLE 1:** Variables description, measurement, and data sources.

Variables	Description	Measurement	Sources
GDP	Carbon dioxide emission	Constant 2015 US$	WDI, World Bank
CO_2_	Non-renewable energy consumption	Million metric tons (Mmt),	WDI, World Bank
TOP	Trade opening	In percent of GDP	WDI, World Bank
RA	Rail infrastructure investment	Constant 2015 US$	OECD database
RO	Road infrastructure investment	Constant 2015 US$	OECD database
AI	Air infrastructure investment	Constant 2015 US$	OECD database

## Methodology and empirical findings

Panel data estimation techniques are often subject to cross-sectional dependencies and can lead to biased hypothesis testing and inference. Therefore, it becomes important to detect cross-sectional dependencies in variable models of panel data (Bilgili et al., 2017; Munir et al., 2020). Hence, the cross-sectional dependence test proposed by Pesaran et al. (2008) is used for this purpose. We explored variable integral properties after an initial cross-sectional dependence analysis by using the cross-sectional ally enhanced Im-Pesaran-Shin (CIPS) unit root test (Pesaran, 2007). Pesaran (2007) augmented the standard Dickey–Fuller test to account for cross-sectional dependencies by taking cross-sectional averages of country-specific data lags. Pesaran estimates an individual cross-section augmented Dickey–Fuller (CADF) statistic by assuming the following regression;


(2) $$\Delta \,{\text{y}}_{\text{it}}=\alpha_{\text{i}}+\delta_{\text{i}}\,y_{\text{i},\text{t}-1}+\phi_{\text{i}}\,{\bar{y}}_{t-1}+\theta_{\text{i}}\,\Delta \,{\bar{y}}_{t-1}+\upsilon_{\text{it}}$$

And it is recommended to test the null hypothesis of the variable with unit root (H0 : δi = 0 for all i) and the alternative hypothesis without the unit root of the variable (H1 : δi < 0). Simple average of individual (CADFi) statistics can be used to estimate standard CIPS statistics;


$$\text{CIPS}=\sum_{i=1}^{N}C\,A\,D\,F_{i}/N$$

After determining the degree of integration of the variables, this study can use Pedroni (1999, 2004) and Kao (1999), to examine the robustness of the estimated results. These two tests are based on the residual-based two-step cointegration test of Engle and Granger (1987). The first residual-based cointegration test proposed by Pedroni (1999, 2004) had a double-ranked cointegration test, called a panel test and a group test. Panel tests include panel ADF-statistic, panel PP-statistic, panel v-statistic and panel rho-statistic. The group test includes the group ADF statistic, the group rho statistic, and the group PP statistic are three statistics. These seven statistics are asymptotically dispersed or distributed by the standard normal and are derived from the following long-term models.


(3) $${\text{Z}}_{\text{it}=}\,\beta_{\text{i}}+\rho_{\text{i}}+\sum_{j=1}^{k}\alpha_{j\,i}\,{\text{X}}_{\text{jit}}+\mu_{\text{it}}$$

where Z and X are the variables for which the first derivative is expected to be integrated.

The article "Empirical analysis of the impact of China–Japan–South Korea transportation infrastructure investment on environmental degradation and the validity of the environmental Kuznets curve hypothesis" was retracted in 2023. Reason: a breach of policy by an author.

The following is the estimated residuals structure.


(4) $$\mu_{\text{it}}=\lambda_{\text{i}}\,\mu_{\text{it}-1}+\varepsilon_{\text{it}}$$

Pedroni (1999, 2004) proposed the null hypothesis that cointegration does not exist between variables and explained the following panel data cointegration system.


(5) $${\text{Z}}_{\text{it}}=\beta_{\text{i}}+\alpha \,X_{\text{it}}+\mu_{\text{it}}$$

The maximum likelihood-based panel cointegration statistic will be compared with the seven panel cointegration tests of this study. According to Uzar (2020), the best attribute to determine long-term relationships is cointegration, group statistics.

Kao’s cointegration technique, developed by Kao (1999), is another test used in this study to determine long-term associations between variables and can be implemented under the assumption of crossed homogeneity coefficients and gives similar results to Pedroni’s test. However, the Kao and Pedroni cointegration tests have the disadvantage of assuming cross-sectional independence and are therefore considered to be the first generation cointegration tests, although these two cointegration tests have been widely used in various literatures. The results of the first-generation cointegration tests were considered invalid because they did not take into account the existence of cross-country dependencies. Thus, this study uses the second-generation cointegration test proposed by Westerlund (2007) that considers the problem of cross-sectional dependence.

After establishing long-term panel cointegration, panel Dynamic Ordinary Least Squares (DOLS) and Fully Modified Ordinary Least Squares (FMOLS) are used to determine the elasticity of the long-term variables.

The FMOLS procedure is the most suitable method to use in the presence of panel data cointegration analysis, which corrects for serial correlation, endogeneity bias, and simultaneous bias (Balsalobre-Lorente and Leitão, 2020; Rahman and Vu, 2020). To check the robustness of the results, the study adopted the DOLS method. Kao and Chiang (2001) suggested that panel DOLS estimator using Monte Carlo outperforms panel FMOLS for small sample sizes because of its out-of-sample properties over panel FMOLS estimators.

The article "Empirical analysis of the impact of China–Japan–South Korea transportation infrastructure investment on environmental degradation and the validity of the environmental Kuznets curve hypothesis" was retracted in 2023. Reason: a breach of policy by an author.

First, the LMadj specification of the cross-sectional dependence test of Pesaran et al. (2008) is used to reveal whether there is cross-sectional dependence in the model and individual data. The findings in Table 2 expressed that null hypothesis of no cross-section dependence for the model is accepted, whereas for the variables, null hypothesis of no cross-section dependence is rejected.

**TABLE 2:** Result of cross sectional dependence test.

Test	InCO2	InGDP	InGDP2	InGDP3	InRA	InRO	InAI	InTOP
LMadj	22.701	21.71	21.83	24.35	6.16	10.02	8.76	0.817
	(0.000)	(0.000)	(0.000)	(0.000)	(0.000)	(0.000)	(0.000)	(0.474)

In parentheses are the probability values, the null hypothesis of the LMadj test shows no cross-sectional dependence.

Therefore, the use of cointegration tests and coefficient estimates is feasible due to the acceptance of the cross-sectional independence explored by the first-generation panel data methods (Pesaran and Tosetti, 2011). A second-generation panel unit root/stationarity approach is now required to determine the level of integration of variables (Dogan and Inglesi-Lotz, 2020; Payne and Apergis, 2021; Yunzhao, 2022).

Due to variable cross-sectional dependencies, we will continue to use the CIPS unit root test. The results in Table 3 report that the null hypothesis for variables with a unit root is accepted, while the alternative hypothesis for variable data without a unit root is accepted after the first differencing. Cointegration among the variables proposed in the model now needs to be explored because the variables have the homogeneous integral property of I(1).

**TABLE 3:** The results of CIPS unit root test.

		LnCO2	lnGDP	lnRA	lnRO	lnAI	lnTOP
Levels	Constant	–1.29	–1.13	–1.61	–2.27	–1.63	–1.98
	Trend + Constant	–2.31	–1.58	–1.70	–1.09	−1.27**	–1.68
First differences	Constant	−3.88***	−2.17***	−3.80**	−4.46***	−4.43***	−5.41***
	Trend + Constant	−3.01***	−2.51***	−3.34***	−4.52***	−4.84***	−4.92***
Critical Values	−2.09 (10%)	2.55(10%)					
	−2.27 (5%)	−2.66(5%)					
	−2.35 (1%)	−2.85(1%)					

*K* = 2 is the maximum lag length chosen. Asterisk ***, **, and * show significance levels of 1, 5, and 10%, respectively.

Long-term cointegration among variables is explored through three cointegration tests by Pedroni (1999, 2004), Kao (1999), and Westerlund (2007), as shown in Table 4. Results that rejected the null hypothesis of no cointegration were approved based on the significance of the three within-dimension statistics and the two between-dimension statistics in the 7-panel cointegration tests. A second test of Kao’s panel cointegration results also suggests a long-term relationship between panel variables, as the ADF statistic is significant at the 1% level.

The article "Empirical analysis of the impact of China–Japan–South Korea transportation infrastructure investment on environmental degradation and the validity of the environmental Kuznets curve hypothesis" was retracted in 2023. Reason: a breach of policy by an author.

**TABLE 4:** The findings of panel cointegration test by Pedroni (1999, 2004), Kao (1999) residual cointegration test, and Westerlund (2007) cointegration test.

	Within-dimension	
	Statistics	*P*-value
Panel v-Statistic	1.89**	0.04
Panel rho-Statistic	0.92	0.95
Panel PP-Statistic	−1.18***	0.00
Panel ADF-Statistic	−3.21***	0.01

	**Between-dimension**	

Group rho-Statistic	1.21	0.89
Group PP-Statistic	−3.16***	0.00
Group ADF-Statistic	−2.27***	0.00
Kao (1999) **residual co-integration test**		
ADF	−3.46***	0.00
Westerlund (2007) **cointegration test**		
Gt	−4.17***	0.00
Ga	−4.58***	0.00
Pt	−15.64***	0.00
Pa	−4.41**	0.03

Asterisks ** and *** indicates 5 and 1% significance level.

The present study also used the Westerlund cointegration test to determine the panel cointegration association among the proposed variables by considering cross-sectional dependencies to test the validity of the former test and thus outperform the first generation cointegration test. The results of the Westerlund cointegration test show that the four test statistics Pa and Pt for panel cointegration, as well as Ga and Gt for individual countries, support the existence of cointegration.

The results of the long-term estimated parameters using Equation 1 are shown in Table 5. The results show that GDP has a significant positive effect, and GDP2 and GDP3 have significant adverse effects on environmental degradation, respectively. These results confirm the validity of the inverted U shaped EKC hypothesis in selected panel of countries. The sign of the GDP coefficient is significantly positive (GDP > 0), GDP2 is significantly negative (GDP2 < 0), and GDP3 is also significantly negative (GDP3 < 0). The positive effect of GDP on environmental degradation persists to a certain extent due to scale effects. Compared to regenerative capacity in earlier stages of economic development, this may improve the use of natural resources, leading to increased greenhouse gas emissions from human activities. The adverse effects of GDP squared and GDP cubed above a certain level are due to technology and compositional effects, which in turn develop clean activities and environmentally friendly technologies. These findings are very much in line with the studies of Gokmenoglu and Taspinar (2018); Sirag et al. (2018), Ganda (2019); Mikayilov et al. (2019), Tzeremes (2019); Adebayo (2020), Alola and Ozturk (2021); Awan and Azam (2021), Minlah and Zhang (2021), and Murshed et al. (2021). Road infrastructure investment (RO) has a significant positive effect, while railway infrastructure investment (RA) has a significant adverse effect on environmental degradation. In this context, for every 1% increase in railway infrastructure investment, the degree of environmental degradation can be reduced by 0.028%, and for every 1% increase in road infrastructure investment, the degree of environmental pollution can increase by 0.06%. This may be due to the scale, cost-effectiveness and cleaner technology of the rail transport system. First, since the end of 1881, the railway industry has made extensive use of electrical power systems (Skjong et al., 2015). Conservative rail systems are no longer common and contain more pollutant-producing technologies than electrical systems. In fact, Gautam et al. (2019) stated that increased investment in rail infrastructure is a precaution against the use of fossil fuel based technologies as more energy efficient and environmentally friendly technologies emerge. Second, rail transportation systems require less land use than road transportation systems, but higher than air transportation systems. This may present an opportunity to maintain a balance between land use and utility creation. Third, the railway industry has huge potential for passenger and freight transport. Rail transport systems with lower emissions and resource usage allow more passengers and freight to be transported. In addition, the economies of scale of the rail industry for passenger and freight transport are likely to be higher than for traditional air or road transport systems.

The article "Empirical analysis of the impact of China–Japan–South Korea transportation infrastructure investment on environmental degradation and the validity of the environmental Kuznets curve hypothesis" was retracted in 2023. Reason: a breach of policy by an author.

**TABLE 5:** The result of estimated parameters by FMOLS and DOLS methods, InCO2 = f (InGDP, InGDP2, InGDP3, InRO, InRA, InAI, and InTOP).

Variables	Panel fully modified ordinary least squares (FMOLS)	Panel dynamic ordinary least methods squares (DOLS)
InGDP	0.536*** (6.532)	1.643*** (5.493)
InGDP^2^	−0.548*** (−6.232)	−1.736*** (−5.204)
InGDP^3^	−0.848*** (−6.235)	0.501*** (5.324)
InRO	0.060***(8.963)	0.045*** (6.518)
InRA	−0.028*** (−5.765)	−0.095*** (−4.849)
InAI	0.050*** (8.963)	0.025*** (6.518)
InTOP	0.187*** (8.963)	0.705*** (6.518)

Asterisk *** indicates statistical significance at 1% level, where inside in the parentheses are t-statistics.

Air infrastructure investment (AI) has a progressive and statistically significant impact on environmental pollution. Every 1% increase in air infrastructure investment stimulates environmental pollution by 0.05%. First, the positive progressive impact of the air transport system on environmental degradation is due to the large amount of land use required to build air transport facilities. In addition, fertile areas and wetlands may be lost as highways, airports and airport transportation networks are built. Deforestation can be increased with higher demand for nature-based building materials (Seddon et al., 2021). Second, aviation, which accounts for nearly 5% of man-made emissions, not only increases carbon emissions and worsens the composition of the atmosphere, but also contributes to air pollution by assimilating necessary ground services with conventional vehicles. Water is also polluted as chemicals and emissions increase. All of these pose significant risks to environmental sustainability and human wellbeing.

The article "Empirical analysis of the impact of China–Japan–South Korea transportation infrastructure investment on environmental degradation and the validity of the environmental Kuznets curve hypothesis" was retracted in 2023. Reason: a breach of policy by an author.

The effect of trade opening (TOP) on environmental degradation is gradual and statistically significant. For every 1% increase in trade openness, environmental pollution will increase by 0.187%. This is related to the failure of the environmental conditions of trade agreements and the aggravating effect of trade liberalization on environmental pollution.

Country wise estimation results by the FMOLS strategy reported in the following Table 6. Country-wise estimates of the carbon-emission-based FMOLS strategy in the model show that GDPs significantly stimulate carbon emissions, while GDP2 and GDP3 significantly reduce carbon emissions in China and South Korea. However, in Japan, GDP and GDP3 have a significantly positive impact on environmental degradation, while GDP2 has a significant negative impact on environmental pollution. This result confirms the validity of the inverted U-shaped EKC hypothesis in China and South Korea, while the N-shaped EKC is only valid in Japan. Road infrastructure investment (RO) has a significant positive effect, while railway infrastructure investment (RA) has a significant adverse effect on environmental degradation in China, Japan and South Korea. Similarly, Air infrastructure investment (AI) and trade opening have had a progressive and statistically significant impact on environmental pollution in China, Japan, and South Korea.

**TABLE 6:** Country-wise results estimated by FMOLS, InCO2 = f (InGDP, InGDP2, InGDP3, InRA, InRO, InAI, and InTOP).

Country	lnGDP	LnGDP^2^	lnGDP^3^	InRA	InRO	InAI	InTOP	R^2^	Adj R^2^
South Korea	0.81 (9.74)***	−0.72 (−8.23)***	−0.48 (−5.97)***	−0.73 (−3.56)***	0.52 (−6.64)***	0.47 (4.23)***	0.06 (5.26)***	0.99	0.98
China	0.43 (4.59)***	−0.37 (−4.24)	−1.48 (−7.92)***	−0.29 (−5.42)***	0.58 (8.38)***	0.15 (5.28)***	0.02 (6.19)***	0.96	0.97
Japan	0.28 (0.97)	−0.86 (−2.86)***	0.75 (2.57)***	0.53 (3.37)***	0.25 (4.87)***	0.25 (4.02)***	0.25 (4.02)***	0.98	0.99

Asterisks *, **, and *** indicate statistical significance at 10, 5, and 1%, respectively. Inside in the parentheses are t-statistics.

The article "Empirical analysis of the impact of China–Japan–South Korea transportation infrastructure investment on environmental degradation and the validity of the environmental Kuznets curve hypothesis" was retracted in 2023. Reason: a breach of policy by an author.

## Conclusion

East Asian countries (China, Japan, and South Korea) have experienced rapid economic growth as a result of industrialization, however, this has had environmental consequences and raised concerns about environmental sustainability. The main purpose of this study is to reveal the environmental impact of infrastructure investment on the transportation systems of selected East Asian countries (China, South Korea, and Japan) that have undergone rapid urbanization due to industrialization and economic growth in the context of the EKC assumption. Also determine which transport investments are environmentally friendly to achieve low pollution goals and ensure the sustainability of urban transport facilities by developing greener transport investment policies and building environmentally friendly transport technologies. First the study detected cross-sectional dependencies in variable models of panel data by Pesaran et al. (2008). The result demonstrated that there is no cross sectional dependence in the model. We explored variable integral properties after an initial cross-sectional dependence analysis by using the cross-section enhanced Im-Pesaran-Shin (CIPS) unit root test (Pesaran, 2007). After determining the degree of integration of the variables, this study used Pedroni (1999, 2004), Kao (1999), and Westerlund (2007) to examine long-term cointegration among variables. After establishing long-term panel cointegration, panel Dynamic Ordinary Least Squares (DOLS) and Fully Modified Ordinary Least Squares (FMOLS) are used to determine the elasticity of the long-term variables. The results show that GDP has a significant positive effect, and GDP2 and GDP3 have significant adverse effects on environmental degradation, respectively. These results confirm the validity of the inverted U shaped EKC hypothesis in selected East Asian countries. Road infrastructure investment (RO) has a significant positive effect, while railway infrastructure investment (RA) has a significant adverse effect on environmental degradation. Air infrastructure investment (AI) has a progressive and statistically significant impact on environmental pollution. Also the effect of trade opening (TOP) on environmental degradation is gradual and statistically significant. Country-wise estimates of the carbon-emission-based FMOLS strategy in the model show that GDPs significantly stimulate carbon emissions, while GDP2 and GDP3 significantly reduce carbon emissions in China and South Korea. However, in Japan, GDP and GDP3 have a significantly positive impact on environmental degradation, while GDP2 has a significant negative impact on environmental pollution. This result confirms the validity of the inverted U-shaped EKC hypothesis in China and South Korea, while the N-shaped EKC is only valid in Japan. Road infrastructure investment (RO) has a significant positive effect, while railway infrastructure investment (RA) has a significant adverse effect on environmental degradation in China, Japan and South Korea. Similarly, Air infrastructure investment (AI) and trade opening have had a progressive and statistically significant impact on environmental pollution in China, Japan, and South Korea.

The article "Empirical analysis of the impact of China–Japan–South Korea transportation infrastructure investment on environmental degradation and the validity of the environmental Kuznets curve hypothesis" was retracted in 2023. Reason: a breach of policy by an author.

If we propose a set of reform policies in the context of EKC, those selected East Asian countries that are on the downhill of EKC will have to change their production techniques and encourage structural transformation of their polluting sectors toward environmental protection. Promoting the development of renewable resources such as wind, wave and solar energy is essential to absorb the adverse externalities of resource use in production and consumption activities and to limit the use of non-renewable resources such as fossil fuels. The selected countries should subsidize private R&D activities to increase the affordability of supply of clean energy and renewable investment projects. Modern rail systems that run on electricity are considered less polluting, so the share of rail infrastructure investment in the transport mix can help build sustainable and safe transport systems at the city Centre and intercity levels and reduce emissions in China, Japan, and South Korea. In addition, policymakers should move away from traditional polluting road and air infrastructure investments and encourage new facilities or retrofit old roads and airports with environmentally friendly building materials. Strict enforcement of the prevailing environmental conditions of trade agreements should be encouraged to reduce the increasing impact of free trade on environmental pollution. In this case, the implementation of such agreements and legislative proposals should be actively monitored by international organizations such as the World Trade Organization. Finally, policymakers should take an active role in implementing the necessary legislation and consider increasing the technological effectiveness of international trade by banning the import of polluting technologies.

This study has certain limitations in terms of data limitations, and we only included data from selected East Asian countries (China, Japan, and South Korea) from 1995 to 2020. The temporal dimension of the data can be expanded in future studies, which will increase the power and scale of the test. In addition, the impact of inland waterway investment on ecological sustainability should be investigated through future research, which was not investigated in this study due to lack of data, which will be a research gap for future studies.

The article "Empirical analysis of the impact of China–Japan–South Korea transportation infrastructure investment on environmental degradation and the validity of the environmental Kuznets curve hypothesis" was retracted in 2023. Reason: a breach of policy by an author.

## Data availability statement

The original contributions presented in this study are included in the article/supplementary material, further inquiries can be directed to the corresponding author.

## Author contributions

AA and YLi contributed to the conceptualization of the study, analysis, design, conclusions, reviewed the manuscript, and approved the final submission. HL, YLu, RT, and YC revised the study, software data curation, editing and literature search. All authors contributed to the article and approved the submitted version.
